# Prevention of Severe Respiratory Tract Infection and Prognosis in Neurosurgical Patients with Severe Tracheotomy Based on 5E Rehabilitation Nursing Model

**DOI:** 10.1155/2022/2727679

**Published:** 2022-07-05

**Authors:** Qing Zhang, Lei Wan, Qin Chen, Chen Li, Ningning Wang, Yang Wang, Yuanyuan Li, Jingjing Huang, Qin Hu

**Affiliations:** Department of Neurosurgery, Zhongnan Hospital of Wuhan University, Donghu Road-169, Wuhan, Hubei Province 430071, China

## Abstract

**Background:**

Continuous nursing based on 5E rehabilitation mode can improve the physiology and psychology of patients to some extent. The purpose of this study was to explore the effect of continuous nursing of 5E rehabilitation mode on the prevention and prognosis of severe respiratory tract infection in patients with severe tracheotomy in neurosurgery.

**Objective:**

To explore the effect of 5E rehabilitation nursing model on the prevention of severe respiratory tract infection and prognosis in patients with severe tracheotomy in neurosurgery.

**Methods:**

The starting and ending time of this study is from February 2019 to July 2021. In this paper, 60 patients with severe tracheotomy were divided into the control group and research group according to random number table method. The former group received routine nursing, and the latter group received rehabilitation nursing model based on 5E. The patients' satisfaction, oxygenation index, partial pressure of carbon dioxide, partial pressure of oxygen, SAS, SDS score, incidence of severe respiratory tract infection, and quality of life scores were compared.

**Results:**

The nursing satisfaction of the research group was higher than that of the control group (*P* < 0.05). 24 hours after weaning, the oxygenation index and partial pressure of oxygen in the research group were higher than those in the control group, while the partial pressure of carbon dioxide in the research group was lower than that in the control group (*P* < 0.05). After nursing, the scores of self-rating anxiety scale and self-rating depression scale in the research group were lower than those in the control group, and the difference was statistically significant (*P* < 0.05). The incidence of severe respiratory tract infection in the research group was significantly lower than that in the control group (*P* < 0.05). After nursing, the scores of physiological function, psychological function, social function, and health self-cognition in the research group were lower than those in the control group (*P* < 0.05).

**Conclusion:**

The nursing program of neurosurgical patients with severe tracheotomy based on 5E rehabilitation model can effectively enhance patients' nursing satisfaction, activities of daily living, anxiety, and depression and promote the prognosis.

## 1. Introduction

In the past 30 years, stroke has become the number one killer affecting our national health [1]. The result of this change is the rapid development of neurosurgery, and neurological severe disease has played a very important role in the development of neurosurgery. Neurocritically ill patients often use artificial airways because of their illness [2]. Generally speaking, patients who may use a ventilator for a long time will undergo tracheotomy. These patients who use ventilator for a long time may reuse the ventilator because of hypoxemia, sputum obstruction of the airway, and other reasons. At present, the weaning failure rate of surgical intensive care unit can be as high as 10% to 19% [3]. As a part of critical medicine, neurological critical disease is also faced with the airway management problems that all critically ill patients will encounter. In general, artificial airway is established because of respiratory insufficiency, airway obstruction, and other reasons [4]. In addition, the indications for the establishment of artificial airway in neurosevere patients are as follows: first, coma caused by craniocerebral injury, cerebrovascular accident, intracranial infection. Glasgow coma score is less than or equal to 8 [5]. Second, severe neurological patients have a decline in their ability to maintain their own airway patency due to disturbance of consciousness and long-term bedridden. For example, patients' ability to cough up sputum is weakened, and it is easy to fall back of the tongue [6]. Thirdly, when the disease affects the respiratory centre (e.g. brain stem haemorrhage, cerebral infarction, brain herniation, etc.) it may cause impairment or even complete destruction of respiratory function. Fourth, when bulbar palsy occurs it can affect the patient's swallowing and coughing functions. Among these neurocritical patients who establish artificial airway, there may be some patients who need to use ventilator for a long time, and in general, tracheotomy is recommended for those who are expected to use ventilator for more than 2 weeks [7]. However, tracheotomy destroys the original physiological structure of the airway and has an impact on the patient's airway management. Airway management in patients with severe neurological diseases is a complex task. Respiratory management is a set of perfect process, from the first step of intraoperative airway management to the final successful removal of mechanical ventilation, all need meticulous management, poor management in the early stage may bring difficulties to oxygen therapy in the later stage and even lead to the reuse of the ventilator, so the early respiratory management will have an important impact on the effect of oxygen therapy in the later stage. Therefore, we should fully understand the particularity of respiratory management in patients with neurological critical illness.

Some scholars have found that neurosurgical patients with severe tracheotomy often have higher demands for perioperative care, and targeted nursing measures will help to prevent the risk of severe respiratory tract infection in such patients. This courage will contribute to the prognosis of patients [8]. The outline of the 2030 year plan for healthy China proposes to adjust and optimize the health service system and strengthen early diagnosis, early treatment, and early rehabilitation. 5E rehabilitation model, as a new nursing model, was put forward by the Life Rehabilitation Advisory Committee of the International Rehabilitation Association in 1994, which is referred to as “5E” in clinic. It includes five parts: encourage, education, exercise, employment, and evaluation. This model emphasizes giving full play to the role of nurses and intervening patients in all aspects of physiology, psychology, and ability from the perspectives of clinical educators, supporters, and coordinators. Research shows that rehabilitation training can promote the rehabilitation of patients, maximize the recovery of residual function, enhance the physical function and psychological state of patients, and improve their ability of life and quality of life [9]. At present, 5E rehabilitation mode has been widely adopted in patients with diabetes, orthopaedics, chronic obstructive pulmonary disease, and dialysis in China. Continuous nursing based on 5E rehabilitation model can improve the physiology and psychology of patients to a certain extent [10]. In this study, it was adopted to prevent severe respiratory tract infection in patients with severe tracheotomy in neurosurgery, aiming to promote the activities of daily life and psychological status of patients with severe tracheotomy in neurosurgery and to evaluate the effect of the nursing program on the prevention of severe respiratory tract infection and prognosis in patients with severe tracheotomy in neurosurgery.

## 2. Patients and Methods

### 2.1. Normal Information

The starting and ending time of this study is from February 2019 to July 2021. In this paper, 60 patients with severe tracheotomy were divided into the control group and research group according to random number table method. The former group received routine nursing, and the latter group received rehabilitation nursing model based on 5E. In the control group, the age ranged from 18 to 68 years, with an average of 51.44 ± 3.64 years old, including 18 males and 12 females. In the research group, the age was 44-76 years, with an average of 51.48 ± 3.42 years old, including 16 males and 14 females. There exhibited no statistical significance in the general data. This study was permitted by the Medical Ethics Association of our hospital, and all patients noticed informed consent. This study is a prospective study. Research samples were randomly assigned to each group.

The inclusion criteria are as follows: (1) age ≤ 70 years and ≥18 years, (2) patients with tracheotomy after neurosurgery, (3) in accordance with the recommendation of the special working group on evidence-based medicine for ACCP/AARC/SCCM offline guidelines, and (4) the patient himself or his legal authorized representative is willing to provide informed consent.

The exclusion criteria are as follows: (1) patients with damaged respiratory center, (2) the end stage of chronic disease, (3) complicated with shock, and (4) lactation or pregnancy.

### 2.2. Treatment Methods

The patients in the control group received routine nursing, including basic nursing, psychological nursing, and health education. These specifically include the following: (1) basic nursing: keep the bed unit clean and tidy during hospitalization; keep the hospital environment quiet and tidy, with appropriate temperature and humidity; timely and accurately implement doctor's orders, seriously formulate nursing plans, and provide appropriate nursing measures for patients; and provide discharge guidance for patients before discharge. (2) Psychological nursing: psychological counseling was given to patients when they were admitted to hospital, psychological support was provided for them, and patients were encouraged to actively cooperate with treatment and nursing. (3) Health education: when the patients were admitted to the hospital, health education was given to the patients and their families, including disease-related knowledge, rational use of drugs, reasonable diet, and adherence to rehabilitation exercise.

The research group accepted the 5E rehabilitation nursing model, and the specific measures were as follows:

1. Encouragement: encourage expression: encourage patients to express their inner thoughts and help once a day according to their psychological condition. Case sharing: share successful treatment cases with patients to encourage patients to actively cooperate with the treatment during hospitalization. Peer encouragement: guide patients in the same ward to encourage each other. When the patients were admitted to the hospital, they should know their psychological status in time and guide them once a week
2. Education: collective health education: focus on health education for patients and caregivers, including disease-related knowledge, rehabilitation, diet, and medication, during hospitalization for 3 times, each time 30~40 min. Individualized guidance: ask patients and caregivers about the content of health education, ask patients questions, give targeted guidance to follow-up after discharge once a week: follow-up by telephone after discharge, urge patients to maintain a healthy lifestyle, pay attention to reasonable diet and emotional control, strictly follow the doctor's advice, follow up regularly, and answer patients' doubts once a week
3. Exercise: turn over: turn over regularly for the patient, once every 2 hours. Good limb position: according to the condition, the patients were placed in supine position, healthy side position, affected side position, bed sitting position, and other positions every 2 hours. Upper limb passive movement: including shoulder joint movement, elbow joint movement, and wrist joint movement. 20~30 min was performed once a day during hospitalization. Passive hand movement: including metacarpophalangeal joint activity and interphalangeal joint activity. Lower limb passive movement: including hip joint movement, knee joint movement, and ankle and foot joint movement. Active exercise: according to the patient's condition, the range of exercise increases gradually, step by step. Bobath handshake was used for upper limb rehabilitation training, and bridge exercise, sitting up and sitting balance training, standing up and standing balance training, and walking training were adopted for lower limb rehabilitation training once a day, each time 20~30 min. Posture transfer: including turning over on bed, movement of lying position on bed, transfer of lying position and sitting position, transfer of sitting position and upright position, and bed-chair transfer. Follow-up after discharge: follow up by telephone after discharge, urge patients to exercise, and answer their doubts once a week
4. Work: ability of daily living training: patients are trained in the ability of daily living, and patients are encouraged to wash their faces and eat as much as possible once a day. Follow-up after discharge: after discharge, the patients were followed up by telephone to know the patients' activities of daily living in time and provide them with individual guidance and advice once a week
5. Evaluation: admission evaluation: general data and basic conditions of patients were investigated. Admission: preintervention evaluation: evaluation of patients' psychological status, physical rehabilitation exercise, daily living ability exercise before intervention, and feedback evaluation of the results. Evaluation of intervention effect: the rehabilitation effect of patients was evaluated

### 2.3. Observation Index

#### 2.3.1. Satisfaction

After consulting the literature and experts' discussion, we designed patients' follow-up satisfaction, a total of 10 items, and recorded patients' satisfaction with follow-up management mode, health education, medical and nursing service, and appointment registration process [11]. It is assigned into four dimensions: very satisfied, satisfied, general, and dissatisfied. Satisfaction rate = very satisfaction rate + satisfaction rate + general rate.

#### 2.3.2. Oxygen Index, Partial Pressure of Carbon Dioxide, and Partial Pressure of Oxygen

The oxygenation index, partial pressure of carbon dioxide, and partial pressure of oxygen at 12 and 24 hours after weaning were calculated.

#### 2.3.3. Psychological Condition

The Hospital Anxiety and Depression Scale (HADS) was jointly developed by Zigmond and Snaith in 1983 for screening anxiety and depression in general hospitals. The scale consists of 14 items and consists of two subscales: anxiety and depression. The score range of each subscale was 0: 21, of which 0: 7 was asymptomatic, 8: 10 was likely to have symptoms, and 11: 21 was positive. Barczak P and Silver Ph found that taking 8 as the critical value had higher sensitivity and specificity. In this study, 8 points were adopted as the screening threshold, and more than 8 points had a positive indication of anxiety/depression. The higher the score, the more serious the degree of anxiety and depression. Cronbach's *α* of the Chinese version of HADS was 0.86, and that of the anxiety and depression subscale was 0.77 and 0.82, respectively, which could be used for the measurement of anxiety and depression in hospitalized patients [12].

#### 2.3.4. Incidence of Severe Respiratory Tract Infection

The incidence of severe respiratory tract infection was calculated.

#### 2.3.5. Quality of Life Scale

The quality of life scale consists of four subscales, including physical, psychological, social, and health self-awareness, with a total of 29 items [13]. Cronbach's *α* coefficient of the scale is 0.79-0.91. The scale was scored by 1-5 grades. The lower the score, the higher the satisfaction.

### 2.4. Statistical Analysis

SPSS26.0 software was adopted for statistical analysis. The measurement data of normal distribution are presented by mean standard deviation ($\bar{x}\pm s$), and the two groups are compared by independent sample *t*-test. The counting data were presented by rate, and the chi-square test was adopted to compare the two groups. *P* < 0.05 indicated that the difference between groups is statistically significant.

## 3. Results

### 3.1. Comparison of Nursing Satisfaction

In the comparison of nursing satisfaction, 23 cases in the research group were very satisfied, 6 cases were satisfied, and 1 case was general, with a satisfaction rate of 100.00%. In the control group, 13 cases were very satisfied, 8 cases were satisfied, 4 cases were general, and 5 cases were dissatisfied; the satisfaction rate was 83.33%. The nursing satisfaction of the research group was higher compared to the control group, and there are statistically significant differences between groups (*P* < 0.05). All the data results are indicated in Figure 1.

### 3.2. Comparison of Oxygenation Index, Carbon Dioxide Partial Pressure, and Oxygen Partial Pressure

In terms of oxygenation index, partial pressure of carbon dioxide, and partial pressure of oxygen, the oxygenation index, partial pressure of carbon dioxide, and partial pressure of oxygen in the research group were lower compared to the control group 12 hours after weaning. 24 hours after weaning, the oxygenation index and partial pressure of oxygen in the research group were higher compared to the control group, while the partial pressure of carbon dioxide in the research group was lower compared to the control group, and there are statistically significant differences between groups (*P* < 0.05). All the data results are indicated in Table 1.

### 3.3. Comparison of Psychological Status

There was no significant difference in psychological status before nursing (*P* > 0.05). After nursing, the SAS and SDS scores of patients decreased. Compared between the two groups, the SAS and SDS scores of the research group were lower compared to the control group, and there are statistically significant differences between groups (*P* < 0.05). All data results are indicated in Table 2.

### 3.4. Comparison of the Incidence of Severe Respiratory Tract Infection

With regard to the incidence of severe respiratory infection, the incidence of severe respiratory infection in the research group was lower compared to the control group, and there are statistically significant differences between groups (*P* < 0.05). All the data results are indicated in Figure 2.

### 3.5. Comparison of Quality of Life Scores

There exhibited no significant difference in the score of quality of life before nursing (*P* > 0.05). After nursing, the scores of quality of life decreased. Compared between the two groups, the scores of physiological function, psychological function, social function, and health self-cognition in the research group were lower compared to the control group, and there are statistically significant differences between groups (*P* < 0.05). All the data results are indicated in Table 3.

## 4. Discussion

Neurological critical patients refer to those critical patients who need intensive care because of craniocerebral trauma, intracranial tumors, intracranial hemorrhage, aneurysms, and other diseases, after or without surgery [13]. Most of these patients have disturbance of consciousness because of their condition, and when patients have disturbance of consciousness, especially when GCS ≤ 8, the ability of spontaneous coughing and sputum is weakened and the root of tongue is more likely to fall back. In addition, brain diseases in specific areas, such as bleeding and tumors, may cause specific functional abnormalities, such as disappearance of swallowing and choking ability and disappearance of spontaneous breathing [14]. Therefore, patients with severe neuropathy should not only deal with primary diseases but also avoid respiratory abnormalities during the recovery of brain diseases; otherwise, they may not only aggravate the primary diseases but also may have diseases of the nervous system that have been controlled but cannot be transferred out of ICU because of abnormalities in the respiratory and circulatory system, prolonging hospitalization and increasing costs [15]. Traditional oxygen therapy is a commonly used method of oxygen delivery, and it is widely used in patients with tracheotomy. However, traditional oxygen therapy has some disadvantages that are not suitable for patients with severe neurotracheotomy, such as low oxygen flow rate, low oxygen temperature, and oxygen dryness. These shortcomings may damage the airway mucosal cilia clearance system of patients, which is not conducive to airway self-discharge [16]. The damaged airway self-purification function is not only more likely to produce sputum scab but also increases the possibility of airway inflammation. The unique physiological effects of high-flow oxygen therapy can make up for the problems existing in ordinary oxygen therapy. First, reducing the ineffective cavity of nasopharynx, transnasal high-flow oxygen therapy can provide airflow up to 60 L/min, so it is difficult to mix air in such high airflow, so as to ensure the oxygen concentration provided, but also wash out the carbon dioxide in nasopharyngeal cavity and reduce the ineffective cavity [16, 17]. Severe neurological patients often need to use a ventilator for a long time because of their primary disease. In this case, many severe neurological patients will undergo tracheotomy, but these long-term ventilator patients will have a high incidence of difficulties in weaning. Of note, in addition to a set of perfect mechanical ventilation management process, oxygen therapy after weaning can also enhance the success rate of weaning. The nervous system and respiratory system affect each other [17]. The effects of the nervous system on the respiratory system are as follows: first, when the patient's disease affects the respiratory center, it can lead to respiratory insufficiency or even complete disappearance; second, when the disease affects the cough function, patients are more likely to have sputum obstruction, pulmonary infection, and other problems; third, when patients have disturbance of consciousness, they may be more likely to fall back of the tongue, and long-term bed rest and lack of exercise may make patients more likely to develop pulmonary infection and diaphragm dysfunction; fourth, mild hypothermia therapy has been used in severe neurological diseases in recent years [18]. Although some literatures have reported that mild hypothermia therapy did not enhance the prognosis of patients, mild hypothermia therapy can protect brain tissue by reducing brain metabolism, protecting blood-brain barrier, reducing brain edema, reducing the production of some toxic products, and promoting brain cell recovery. But inevitably, mild hypothermia therapy also has some disadvantages, such as hypothermia will increase the risk of infection, and this infection is likely to be pulmonary infection [19]. The effects of the respiratory system on the nervous system are as follows: first, the central system is extremely sensitive to hypoxia, which may aggravate the original condition in patients with central injury; second, the effect of partial pressure of carbon dioxide on cerebral vessels and the decrease of partial pressure of carbon dioxide during hyperventilation can reduce cerebral blood flow and reduce intracranial pressure, but it may also cause cerebral ischemia and aggravate the patient's condition; third is the setting of positive end-expiratory pressure (PEEP). It is believed that PEEP exceeding 15cmHO will increase intrathoracic pressure, affect intracranial blood flow reflux, and increase intracranial pressure [20].

Patients with severe neuropathy often need to establish artificial airways because of the change of consciousness, sedation therapy, and the weakening of swallowing and choking ability [21]. And some of these patients need long-term mechanical ventilation for the same reason, but mechanical ventilation is a process of treatment and a means of treating patients with respiratory insufficiency, not the purpose of treatment. The purpose of treatment is to enable patients to get out of the ventilator and breathe independently. The shorter process, the better outcomes. Because of the extension of mechanical ventilation, there will be a series of problems such as lung infection, decreased diaphragm function and psychological dependence on ventilator [21, 22]. When a patient has a pulmonary infection, it may first aggravate the patient's condition, and the consumption caused by the infection will make the patient's nutritional status even worse. Once the infection is not controlled in time, it will progress to septic shock. It will also make the patient's circulatory system disorder; at this time, in order to ensure the blood supply to the brain and other important organs of the body, vasoactive drugs will have to be used. If the vasoactive drugs are used for a long time, it will affect the peripheral circulation of the patients, reduce the urine volume of the patients, and enter a vicious circle that is difficult to control, even if the timely control of pulmonary infection does not cause septic shock, but it will still cause fever, increased respiratory secretions, and increased airway resistance, making it difficult for patients to wean. The decline of diaphragm function is the decline of respiratory muscle function of patients; diaphragm is the most important respiratory muscle, so diaphragm dysfunction will directly lead to respiratory disorders, making patients weaning failure. The psychological dependence on ventilator will make patients recover the function of spontaneous breathing in time and cannot be weaned smoothly, which will not only cause additional costs but also waste medical resources, so other patients in need of treatment cannot get timely treatment. Moreover, the incidence of acute respiratory failure caused by changes in consciousness and other reasons in patients with severe neuropathy is as high as 50% to 80% [22]. Therefore, the respiratory management of patients with severe neuropathy is particularly important. First of all, due to the change of consciousness and sedation therapy, patients' spontaneous breathing may be impaired in varying degrees, which may lead to long-term mechanical ventilation, but studies have indicated that mechanical ventilation time ≥ 7 days is an independent risk factor for ventilator-associated pneumonia (VAP). Patients with long-term mechanical ventilation may have selective tracheotomy, and tracheotomy is also a risk factor for VAP [23]. Once the patient has VAP, it may concentrate the patient's condition, prolong the ventilation time, and prolong the ICU hospitalization time of the patient. Long-term mechanical ventilation may not only lead to VAP but also mechanical ventilation-related diaphragmatic dysfunction (VIDD), and it is a part of acquired weakness (ICUAW) in intensive care unit, which is caused by neuromuscular weakness caused by multiple organ dysfunction and long-term immobilization in patients treated with ICU for a long time in recent years [24]. Compared with other muscles, the diaphragm is more prone to dysfunction, which makes weaning more difficult [25]. According to the current research, VIDD may occur at 18-24 hours [26, 27]. The longer thinning diaphragm is more obvious, having the average daily reduction of 6% [28]. Therefore, the longer the time of mechanical ventilation, the worse the diaphragm function of patients, and early weaning can improve the diaphragm function of patients [29]. Weaning is not the sooner the better, because the effect of mechanical ventilation on the diaphragm is comprehensive, not only in diaphragm thickness but also in diaphragm blood flow, mitochondria, protein, and enzyme synthesis [30]. Although a large number of studies have indicated that long-term mechanical ventilation is disadvantageous to patients, weaning should ensure the recovery of patients' autonomous respiratory function. The condition has reached the index of weaning; otherwise, blind weaning not only cannot benefit the patient but may reduce the blood oxygen saturation of the patient and even lead to circulatory instability.

There are more cases of long-term mechanical ventilation in patients with severe neurological diseases, and long-term mechanical ventilation will lead to VAP and VIDD, making it difficult to weaning [31]. For neuropathic severe patients with tracheotomy, weaning is also difficult because of sputum scab formation, which is more likely to occur in patients with tracheotomy, because tracheotomy not only destroys the physiological structure of the airway but also shortens part of the airway, weakening the function of the airway to heat and humidify the gas. It also makes it easier for sputum scabs to form, causing airway obstruction and difficulty in breathing. In addition to the management of respiratory system, circulation, nutrition, and rehabilitation will affect patients' breathing, good circulation will have a positive impact on patients' breathing, and cardiogenic pulmonary edema and pleural effusion will have a direct impact on patients' respiration. And patients with unstable circulatory function may not be able to wean, prolonging the time of mechanical ventilation. A more common situation is that the patient is mechanically ventilated for a long time and has mechanical ventilation-related pulmonary infection, and because of the existence of endotracheal intubation, antibiotics may not be able to achieve good results, so septic shock occurs, resulting in circulatory problems. For patients with severe neurological diseases, it is necessary to ensure adequate brain blood supply, and circulatory instability may lead to insufficient cerebral blood supply. It is disadvantageous to the recovery of the patient's disease and may even cause ischemic cerebral infarction and aggravate the patient's condition, so we must pay attention to the cerebral perfusion pressure of the severe neurological patients. When the patient fluctuates along the bad, we need to be able to deal with it quickly and timely [32]. In the aspect of nutrition, some studies have pointed out that the nutritional status of patients is poor, and low albumin is one of the many factors, which lead to weaning failure, especially when patients have infection, fever, and increased consumption, so it is necessary to adjust the nutrition program. A reasonable nutrition program is very important to the recovery of the patient's condition, that is, to meet the patient's nutritional needs and avoid the patient's low albumin. It is also necessary to avoid the burden of too much diet on the digestive system and cause diarrhea in patients [33]. Patients' long-term disturbance of consciousness and braking will lead to muscle atrophy, lower limb thrombosis, and other problems. Rehabilitation exercise into the critical medicine department can not only help patients alleviate muscle atrophy, lower limb thrombosis, and other problems. It may also enhance the immune function and respiratory function of patients [34].

5E rehabilitation model, as a new nursing model, was put forward by the Life Rehabilitation Advisory Committee of the International Rehabilitation Association in 1994, which is referred to as “5E” clinically. It includes five parts: encourage, education, exercise, employment, and evaluation [35]. Encouragement is psychological intervention to patients, so as to enhance their confidence in overcoming the disease and alleviate their negative emotions. Education is a complete health education for patients to enhance their awareness and awareness of disease knowledge. Exercise is guided by a series of standardized rehabilitation training programs to enhance patients' quality of life and promote their motor function. Work is to enhance the ability of daily life of patients, encourage patients to actively participate in daily life activities, and help patients improve their ability to take care of themselves. The purpose of evaluation is to evaluate the nursing work, analyze the reasons for those with unideal effect, and revise and perfect the nursing plan. This model emphasizes giving full play to the role of nurses and intervening patients in all aspects of physiology, psychology, and ability from the perspectives of clinical educators, supporters, and coordinators. The nursing program in this study was constructed based on the 5E rehabilitation model, which is very mature and widely adopted in clinical practice [36]. Some scholars have pointed out that applying the 5E-based rehabilitation model to patients with severe tracheotomy in neurosurgery can effectively promote the patients' daily life ability [37]. The application of this theory can give full play to the subjective initiative of patients. The actual situation of the patient provides individualized care measures. In this study, 5E rehabilitation model was applied to patients with severe tracheotomy in neurosurgery, starting from five aspects of encouragement, education, exercise, work, and evaluation, to provide individualized rehabilitation nursing measures for patients according to their condition and self-care ability. Therefore, the scheme is feasible on the theoretical level [38]. Through the literature research, the rehabilitation nursing intervention methods for patients with severe tracheotomy in neurosurgery were summarized, and the clinical experts in related research fields were consulted to enhance the nursing plan so as to lay the foundation for the implementation of the program. Therefore, the application of the content of the nursing scheme is feasible [39–41]. There are some limitations in this study. First, the sample size of this study is not large and it is a single-center study, so bias is inevitable. In future research, we will carry out multicenter, large-sample prospective studies, or more valuable conclusions can be drawn.

In summary, 5E rehabilitation model is an effective nursing concept, and the nursing model based on it is of great significance for patients with severe tracheotomy in neurosurgery. The nursing program can effectively improve patients' activity ability and living standards, reduce patients' negative mental state, and improve patients' nursing satisfaction, which is worth popularizing.

## Figures and Tables

**Figure 1:** Comparison of nursing satisfaction between two groups.

**Figure 2:** Comparison of the incidence of severe respiratory tract infection between two groups.

**Table 1:** Comparison of oxygenation index, partial pressure of carbon dioxide, and partial pressure of oxygen between the two groups ($\bar{x}\pm s$).

Group	*N*	Oxygenation index		Partial pressure of carbon dioxide		Oxygen partial pressure	
		After offline 12 h	After offline 24 h	After offline 12 h	After offline 24 h	After offline 12 h	After offline 24 h
C group	30	395.94 ± 23.44	336.49 ± 42.11	36.97 ± 3.31	35.19 ± 2.45	141.29 ± 31.33	125.92 ± 34.23
R group	30	351.29 ± 35.22	394.19 ± 23.11	33.59 ± 1.24	32.10 ± 1.21	133.49 ± 23.34	151.34 ± 34.32
*t*		5.780	6.579	5.237	6.193	2.441	2.872
*P*		<0.01	<0.01	<0.01	<0.01	<0.01	<0.01

**Table 2:** Comparison of psychological status between the two groups ($\bar{x}\pm s$, points).

Group	*N*	SAS		SDS	
		Before nursing	After nursing	Before nursing	After nursing
C group	30	59.82 ± 4.31	47.49 ± 2.67	54.19 ± 3.11	49.53 ± 3.55
R group	30	59.83 ± 4.44	40.91 ± 2.31	54.79 ± 2.56	43.19 ± 2.34
*t*		0.008	10.207	0.815	8.167
*P*		>0.05	<0.01	>0.05	<0.01

**Table 3:** Comparison of quality of life scores between the two groups before treatment ($\bar{x}\pm s$, points).

Group	*N*	Physiological function		Psychological function		Social function		Healthy self-cognition	
		Before nursing	After nursing	Before nursing	After nursing	Before nursing	After nursing	Before nursing	After nursing
C group	30	15.84 ± 4.91	13.86 ± 2.95^a^	16.94 ± 3.91	14.85 ± 4.86^a^	18.82 ± 3.95	16.37 ± 2.81^a^	15.98 ± 3.91	13.86 ± 1.85^a^
R group	30	15.96 ± 4.52	11.84 ± 2.91^b^	16.95 ± 3.86	12.81 ± 1.85^b^	18.84 ± 3.55	12.84 ± 3.81^b^	15.87 ± 3.66	10.83 ± 2.91^b^
*t*		0.098	2.670	0.009	2.148	0.020	4.084	0.112	4.812
*P*		0.921	0.009	0.992	0.035	0.983	<0.01	0.910	<0.01

Note: comparison before and after nursing in the control group, ^a^*P* < 0.05. Comparison before and after nursing in the research group, ^b^*P* < 0.05.

## Data Availability

The datasets used and analyzed during the current study are unavailable due to the patient privacy.

## References

[1] Dong M., Zhou Y., Yang J., Yang J., Liao X., Kang Y. (2019). Compare the effect of noninvasive ventilation and tracheotomy in critically ill mechanically ventilated neurosurgical patients: a retrospective observe cohort study. *BMC Neurology*.

[2] Samra S., Schroeder J. W., Valika T., Billings K. R. (2018). Tracheotomy for difficult airway foreign bodies in children. *Otolaryngology–Head and Neck Surgery*.

[3] Trouillet J. L., Collange O., Belafia F. (2018). Tracheotomy in the intensive care unit: guidelines from a French expert panel. *Annals of Intensive Care*.

[4] Sørensen R. M., Christian G., Thomas H. (2018). National changes in pediatric tracheotomy epidemiology during 36 years. *European Archives of Oto-Rhino-Laryngology: Official Journal of the European Federation of Oto-Rhino-Laryngological Societies (EUFOS): Affiliated with the German Society for Oto-Rhino-Laryngology-Head and Neck Surgery*.

[5] Russell C. J., Thurm C., Hall M., Simon T. D., Neely M. N., Berry J. G. (2018). Risk factors for hospitalizations due to bacterial respiratory tract infections after tracheotomy. *Pediatric Pulmonology*.

[6] Passias A., Margaritis A., Liarmakopoulou A., Tzimas P., Papadopoulos G. (2018). The first case of tracheotomy published in Greece in the 19th century. *Hellenic Journal of Surgery*.

[7] Lugo Machado J. A., Escobedo Delgado H., Mávita Corral C. J. (2017). Tracheotomy in a tertiary health care unit in northwestern Mexico: description and analysis of a series of cases. *Horizonte Médico (Lima)*.

[8] Aydin E., Erol O. (2017). Suprastomal granulation tissue and pediatric tracheotomy decannulation. *Trends in Anaesthesia and Critical Care*.

[9] Wang H. F., Yu L. L., Ruan H., Hu J. L., Yuan W. J., Hao G. H. (2017). Establishment of an evidence-based protocol for tracheotomy care in adult patients. *Shanghai kou qiang yi xue = Shanghai journal of stomatology*.

[10] (2017). Science; studies from West China Hospital provide new data on science (the application of the modified surgical wound dressing in wound care after tracheotomy). *Science Letter*.

[11] Grønhøj C., Charabi B., Buchwald C. V., Hjuler T. (2017). Indications, risk of lower airway infection, and complications to pediatric tracheotomy: report from a tertiary referral center. *Acta Oto-Laryngologica*.

[12] (2017). Surgery-tracheotomy; recent findings from Hiroshima University provides new insights into tracheotomy (prevalence of tracheotomy and percutaneous endoscopic gastrostomy in patients with Guillain-Barr, syndrome). *Biotech Week*.

[13] Wang D., Su L., Han Y. (2017). Direct intralesional ethanol sclerotherapy of extensive venous malformations with oropharyngeal involvement after a temporary tracheotomy in the head and neck: initial results. *Head & Neck*.

[14] Wang Q., Liu Y. H., Wu K. L. (2017). The application of high tracheotomy in forced posture. *Lin chuang er bi yan hou tou jing Wwai ke za zhi =Journal of clinical otorhinolaryngology, head, and neck surgery*.

[15] (2016). Tracheotomy in a critically ill patient: 25 years experience in the pediatric intensive care unit. *Archivos de Pediatría del Uruguay*.

[16] Tsoucalas G. (2016). Theodoros Aretaios (1829-1893) the most eminent surgeon of his era and the first pediatric tracheotomy due to laryngeal diphtheria in modern Greece. *Journal of Universal Surgery*.

[17] Ritchie Rodger T. (1926). Tracheotomy in tuberculous laryngitis. *Proceedings of the Royal Society of Medicine*.

[18] Thomson S. (1918). Tooth impacted in a secondary bronchus of the left lung; removal by tracheotomy and lower bronchoscopy after two unsuccessful attempts by upper bronchoscopy. *Proceedings of the Royal Society of Medicine*.

[19] Redel A., Ritzka M., Kraus S. (2016). Extracorporeal CO_2_ removal as an alternative to tracheotomy in a patient with extubation failure. *Der Anaesthesist*.

[20] Buiret G., Gautheron L., Labrosse-Canat H. (2015). Tracheotomy/tracheostomy management at home and in care centers. *Archives of Otolaryngology and Rhinology*.

[21] Lazarus Medical L. L. C. (2016). Patent issued for ventilator to tracheotomy tube coupling (USPTO 9468730). *Journal of Engineering*.

[22] (2016). Patents; "speech valve for persons having undergone a laryngectomy or tracheotomy" in patent application approval process (USPTO 20160242900). *Politics & Government Week*.

[23] Rolleston J. D., Mac Pherson D. G. (2021). Tracheotomy in an adult for Å’dematous laryngitis in scarlet fever. *Proceedings of the Royal Society of Medicine*.

[24] Thomson S. C. (2019). Papilloma of the larynx in a boy aged 612, of four years' duration, cured by tracheotomy and repeated operations by direct laryngoscopy. *Proceedings of the Royal Society of Medicine*.

[25] (2016). Event horizon limited; researchers submit patent application, "emergency tracheotomy device", for approval (USPTO 20160184543). *Politics & Government Week*.

[26] Liu L. X., Li J. D., Luo X. Z., Chi R. B. (2016). Treatment experience on ICU patients with percutaneous dilational tracheotomy and subsequent delayed bleeding. *Zhonghua er bi yan hou tou jing wai ke za zhi =Chinese journal of otorhinolaryngology head and neck surgery*.

[27] Collins C. G. (2016). Rationale and value of tracheotomy in severe preeclampsia and eclampsia. *Postgraduate Medicine*.

[28] Ruf K., Hackenberg S., Kraus F. (2016). Carbon dioxide laser cordotomy as possible alternative for tracheotomy in a neonate with idiopathic bilateral vocal fold paralysis. *Klinische Padiatrie*.

[29] Narayanan M. K., John Martin K. D., Bhowmik T. (2016). Tracheotomy for management and surgical retrieval of granite stone in a pup. *Intas Polivet*.

[30] Su X., Li Z., Wang M. (2016). The protective effect of different airway humidification liquids to lung after tracheotomy in traumatic brain injury: the role of pulmonary surfactant protein-A (SP-A). *Gene*.

[31] Hassanein A. G., Mabood A. M. A. A. (2016). Can submandibular tracheal intubation be an alternative to tracheotomy during surgery for major maxillofacial fractures?. *Journal of Oral and Maxillofacial Surgery*.

[32] Johan U., Jonas K., Gregori M. (2016). A new safe and cost-effective percutaneous dilatational tracheotomy: safe trach. *Acta Oto-Laryngologica*.

[33] Singh B. S. (2016). In reference to late tracheotomy is associated with higher morbidity and mortality in mechanically ventilated patients. *The Laryngoscope*.

[34] Farida J. P., Lawrence L. A., Svider P. F. (2016). Protecting the airway and the physician: aspects of litigation arising from tracheotomy. *Head & neck*.

[35] Work W. P., Smith M. F. W. (2016). Tracheotomy. *Postgraduate Medicine*.

[36] Stutsman A. C. (2016). Technic of tracheotomy. *Postgraduate Medicine*.

[37] Pan L., Guo Y. (2016). Effect of early versus late tracheotomy in critically ill patients: a systematic review and meta-analysis. *Chest*.

[38] Panchal N., Zide M. (2016). The parkland 12-minute checklist tracheotomy. *Journal of Oral and Maxillofacial Surgery*.

[39] Turković T. M., Lukić A., Pažur I., Ožegić O., Obraz M. (2016). Effect of tracheotomy on clinical course of ventilator-associated pneumonia. *Acta Clinica Croatica*.

[40] Magdić T. T., Anita L., Mladen P. (2016). Comparison of early and late percutaneous tracheotomy in critically ill patients: a retrospective single-center observational study. *Acta Clinica Croatica*.

[41] Bergeron M., Audet N. (2016). One hundred twelve patients above 75 years old with tracheotomy: discharge delayed by 13 days: our experience. *Clinical Otolaryngology*.

